# TNFAIP6 Promotes Gastric Carcinoma Cell Invasion via Upregulating PTX3 and Activating the Wnt/*β*-Catenin Signaling Pathway

This article has been retracted.

**DOI:** 10.1155/2022/5697034

**Published:** 2022-07-06

**Authors:** Hongquan Cui, Ling Zhang, Bin Chen, Fengchun Zhang, Haiyan Xu, Guixiang Ma, Longnv Cao, Miao Wang

**Affiliations:** ^1^Oncology Department Suzhou Kowloon Hospital, Shanghai Jiaotong University School of Medicine, Suzhou 215127, China; ^2^Oncology Department, Siyang Hospital, Suqian 223798, China

## Abstract

Tumor metastasis is a fundamental cause of the poor prognosis of gastric carcinoma (GC). In order to study the problems affecting metastasis and recurrence of gastric cancer, the paper expose that TNF alpha induced protein 6 (TNFAIP6) is aberrantly overexpressed in GC, and patients with high-TNFAIP6 levels exhibited inferior overall survival. Mechanistically, overexpression of TNFAIP6 raised *β*-catenin ectopic nuclear distribution and activated the Wnt/*β*-catenin signal pathway. The experimental results show that TNFAIP6 facilitates the aggressive potential of GC cells through modulating PTX3 expression.

## 1. Introduction

Notable progress has been achieved in gastric carcinoma (GC) therapy. However, metastasis and recurrence of GC still profoundly influence patients' outcomes. A flurry of recent studies illuminating the molecular landscape of GC have identified crucial genomic changes that facilitate the progression of the disease [1, 2]. As metastasis starts with an invasion of the tissue surrounding the primary tumor, it is essential to prevent the invasive cancer cell from moving through the extracellular matrix (ECM), which could serve as an intrinsic barrier to the invasion of metastatic cancer cells [3, 4]. Cancer cells acquire migratory and invasive capacity through altering their genes expressions during the epithelial-to-mesenchymal transition (EMT) process, and the EMT has a profound effect on cancer metastasis [5]. Aberrant expression of TNF*α* stimulated gene-6 (TNFAIP6) has been confirmed to be associated with various human diseases, including tissue injury, malignancies, cardiovascular diseases, and inflammatory conditions [6–8]. TNFAIP6 high-expression predicted poor overall survival in patients with head and neck cancer (HNC) and urothelial carcinomas [9, 10]. In gastric cancer, TNFAIP6 promotes invasion and metastasis of carcinoma cells and indicates a poor prognosis in patients [11]. In addition, TNFAIP6 is upregulated in GC compared with normal tissue and can potentially be applied to blood-based detection assays [12]. However, the biological significance of TNFAIP6 in GC has not been investigated. In this study, we confirm that TNFAIP6 expression is closely related to the poor prognosis of patients with GC. Gain- and loss-of-function experiments manifested that TNFAIP6 is critical in GC cell invasion and EMT process. Our study, for the first time, elucidates the prognosis significance and regulatory mechanism of TNFAIP6 in GC.

The rest of this paper is organized as follows: Section 2 discusses relevant literature and comparative analysis, followed by the clinical treatment methods and evaluation indicators in Section 3. The comparative analysis and data statistics in Section 4.  Section 5 concludes the paper with summary and future research directions.

## 2. Relevant Literature and Comparative Analysis

TNFAIP6 is a member of the hyaluronic-binding protein family, which is involved in extracellular matrix stability and cell migration [13–15]. Previous research underlines the criticality of TNFAIP6 in cancer invasion, metastasis, and prognosis [16, 17]. High TNFAIP6 expression is associated with lymph node metastasis and worse prognosis in patients with gastric cancer, indicating that TNFAIP6 may act as a prognostic marker for gastric cancer. In colon carcinoma, a better clinical outcome is predicted with a lower level of TNFAIP6 [18]. Although the studies reveal some interesting findings regarding TNFAIP6 in cancers, the molecular mechanism of TNFAIP6-mediated GC progression remains elusive.

Here, a striking upregulation of TNFAIP6 expression in GC and elaborated on the biological significance of TNFAIP6 in GC prognosis and progression are observed in this paper. Consistent with previous studies, high TNFAIP6 expression is associated with a worse prognosis in patients with GC. Local and systemic metastasis is a major contributor to dismal prognosis in GC [19]. Next, the phenotypic changes in GC cells caused by the alteration of TNFAIP6 expression are investigated. Gain- and loss-of-function studies provide direct evidence that TNFAIP6 is an essential prometastatic factor. Upon activation, the Wnt/*β*-catenin signal pathway facilitates GC growth and metastases [20]. It is found that TNFAIP6 promotes *β*-catenin accumulation in the nucleus, suggesting that TNFAIP6 activates Wnt signaling. The luciferase reporter gene assay further corroborated that TNFAIP6 had driven the Wnt/*β*-catenin signaling pathway.

By analyzing the gene correlation (string), we can get the coexpression of TNFAIP6 and PTX3. Coincidentally, the contribution of PTX3 in EMT of other types of tumors has been established [21]. This prompt us to speculate whether TNFAIP6 exerts its procancer effect, at least in part, by modulating PTX3. This hypothesis is confirmed by the following: firstly, TNFAIP6 positively regulated PTX3 expression in GC cells. Secondly, the rescue experiment confirm that PTX3 is involved in TNFAIP6-mediated GC cell invasion and EMT. Regrettably, the exact mechanism by which TNFAIP6 protein regulates PTX3 expression is still not clear. The regulation mechanisms at the transcriptional or post-transcriptional need to be identified. Besides, further studies will be needed to clarify the correlation between TNFAIP6 expression and PTX3 expression in patients with GC.

## 3. Clinical Treatment Methods and Evaluation Indicators

### 3.1. GC Tissues

Thirty-four pairs of paraffin-embedded GC tissues and matched paracancerous tissues were purchased from Xian Ailina Biotechnology. The clinical characteristics are provided in Table 1. Informed consent from all participants is obtained. The study protocol is granted by the ethical committee. Immunohistochemistry analysis is performed according to the standard protocol as previously described.

### 3.2. Cell Lines and Immunoblotting

GC cells (SGC7901, MGC803, MKN45 and MKN28) and the gastric epithelial cell line GES-1 are purchased from ATCC (Rockville, USA). Cells are cultured in Dulbecco's modified Eagles medium (DMEM)(Invitrogen, Carlsbad, CA, USA) and 10% fetal bovine serum (FBS) (Invitrogen) supplemented with 1% penicillin-streptomycin (Invitrogen) at 37°C under 5% CO_2_. Total proteins in cells are prepared using RIPA lysis buffer (Beyotime, Nanjing, China). The immunoblotting assay is performed with antibodies against TNFAIP6 (Proteintech Group, IL, USA), *β*-catenin (Proteintech), N-Cadherin (Proteintech), PTX3 (Proteintech), E-Cadherin (Proteintech), Lamin B1 (Proteintech), and GAPDH (Bioworld Technology) as previously described. Nuclear and cytoplasmic fractions are separated using a KeyGEN nuclear and cytoplasmic protein extraction kit (KeyGEN BioTECH, Nanjing, China). Secondary antigoat antibodies are purchased from Beyotime Biotechnology (Nanjing, China).

### 3.3. Vectors and Transfection

2 × 10^5^ SGC7901 or MGC803 cell suspension is seeded in 6-well dishes and grown overnight. Cells are transfected with TNFAIP6 siRNA (si-TNFAIP6, Santa Cruz Biotechnology) using Lipofectamine 3000 (Invitrogen). Negative-control siRNA is used as a siRNA control (si-Con). 48 h post-transfection, cells are harvested and subjected to experiments. The cDNA encoding PTX3 or TNFAIP6 is PCR-amplified using Q5 High-Fidelity DNA Polymerase (New England Biolabs, Ipswich, MA) and inserted into the pcDNA3 vector (Invitrogen), named OE-PTX3 or OE-TNFAIP6, respectively. An empty pcDNA3 vector is utilized as a control. 48 h post-transfection, cells are harvested and subjected to experiments. Stable TNFAIP6 knockdown in SGC7901 cells is established by transfection of shRNA. Briefly, a MISSION® pLKO-empty vector or a vector encoding pLKO-shRNA against TNFAIP6 (Sigma-Aldrich, Inc., MO, USA) are transfected into SGC7901 cells with lipofectamine 3000. TNFAIP6 stable knockdown SGC7901 cells are screened with 1 *μ*g/ml puromycin (Sigma-Aldrich).

### 3.4. Luciferase Reporter Assay and Cell Viability

SGC7901 or MGC803 cell is transfected with TOP-flash or FOP-flash reporter plasmid (Sigma-Aldrich) together with pRL-TK Renilla plasmid (Promega, Madison, WI, USA) with Lipofectamine 3000. 48 h post-transfection, luciferase activity is measured with a dual-luciferases reporter assay kit (Promega). Cell viability is measured using CellTiter 96 aqueous one solution cell proliferation assay (MTS) (Promega). SGC7901 or MGC803 cell is seeded in 96-well plates overnight. At various time points, 20 *μ*l of reagent are pipetted into each well. After 2 h, the absorbance value is assessed at 490 nm under a microplate reader (BioTek Instruments, Colmar, France).

### 3.5. Assay and Cell Invasion

SGC7901 or MGC803 cell (1 × 10^3^ cells/well) is cultured in 6 well plates. Cells are cultured for 2 weeks, and the medium is changed every 3 days. Then, cells are fixed in 10% paraformaldehyde for 15 min followed by staining with 1% crystal violet for 15 minutes.

Cell invasion is measured by bio coat chambers (BD Biosciences, NJ, USA) with polycarbonate membrane filters (8 *μ*m pore size). Cells (5 × 10^4^/well) are plated into the upper chamber, and the lower chamber is filled with a complete medium. After 24 h, the invaded cells are fixed with 4% paraformaldehyde for 10 minutes and dyed with 1% crystal violet for 15 minutes. The number of invading cells is counted under an inverted microscope in 3 random fields.

### 3.6. In Vivo Metastasis Assay

For metastasis assay *in vivo*, sh-NC or sh-TNFAIP6-transfected SGC7901 cells (5 × 10^6^) are injected into the tail vein of nude mice to construct the lung metastasis model (*n* = 4 in each group). After implantation for 35 days, the lungs are harvested for hematoxylin and eosin (H&E) staining. Then, the number of metastatic nodules is calculated in the tissue section. The study protocol is granted by the ethical committee.

### 3.7. Statistical Analysis

Statistical analyses are calculated by using GraphPad Prism 8 (GraphPad, USA). Data are presented as the Mean ± SD. Comparisons between different groups are analyzed by means of paired Student's *t*-test. *P* < 0.05 is statistically significant.

## 4. Comparative Analysis and Data Statistics

### 4.1. TNFAIP6 is Upregulated in GC

To detect the expression of TNFAIP6 in GC tissues, we need to get the mRNA level of TNFAIP6 in 31 pairs of GC specimens and paracancerous tissues. The results of qRT-PCR show that TNFAIP6 expression is obviously increased in GC tissues, as shown in Figure 1. In addition, the IHC assay also indicates that the level of TNFAIP6 is higher in GC tissues than that in paracancerous tissues. Moreover, the prognostic analysis result shows that GC patients in the low TNFAIP6 expression group have a better prognosis than those in the high-expression group. When comparing the gastric epithelial cell line GES-1, GC cells (SGC7901, MGC803, MKN45, and MKN28) exhibit higher TNFAIP6 expression. These data suggest that TNFAIP6 protein is highly expressed in GC.

### 4.2. TNFAIP6 Contributes to GC Cell Growth and Invasion

The role of TNFAIP6 in GC cells growth and invasion are as follows: SGC7901 or MGC803 cell is transfected with TNFAIP6 siRNA (si-TNFAIP6) or corresponding nonsilencing-siRNA (si-Con). Western blot analysis is performed to evaluate knockdown efficiency of endogenous TNFAIP6, as shown in Figure 2. TNFAIP6 knockdown caused profound growth inhibition in GC cells. It shows that TNFAIP6 deletion tremendously suppressed GC cell invasion.

To confirm the above findings, we can get the overexpression of TNFAIP6 in MKN45 cells by transfecting the TNFAIP6 plasmid, as shown in Figure 3. Conversely, the increased expression of TNFAIP6 promote MKN45 cell growth and invasion ability. Altogether, these observations strongly suggest that TNFAIP6 contributes to GC cell migration and invasiveness.

### 4.3. TNFAIP6 Promotes GC Cells EMT

Since an EMT-like process has been associated with GC metastasis, TNFAIP6 promotes EMT, which is examined. Repression of E-cadherin expression and upregulation of N-cadherin are the critical events in EMT induction and cancer metastasis [22].  Figure 4 shows the overexpression of TNFAIP6 increased N-cadherin expression and suppressed E-cadherin expression. TOP/FOP luciferase activity assay exhibited that the canonical Wnt-signaling pathway is activated upon TNFAIP6 overexpression. *β*-catenin nuclear translocation is the marker for Wnt/*β*-catenin pathway activation, and immunoblotting analysis showed TNFAIP6 elevated *β*-catenin levels in the nucleus. String Bioinformatics software is used to predict the coexpressed proteins for TNFAIP6 [23]. In the String coexpression analysis, PTX3 ranked first with a score of 0.988. Excitingly, PTX3 overexpression accelerates hepatocellular carcinoma cell metastasis by enhancing EMT [24]. PTX3 likely mediates the effects of TNFAIP6 on the EMT process in GC. As expected, the silencing of TNFAIP6 efficiently reduced the mRNA level of PTX3 in GC cells.

### 4.4. TNFAIP6-Mediated EMT Process Requires PTX3

To confirm the above results, reintroduce PTX3 in the TNFAIP6 knockdown GC cell, as shown in Figure 5. The knockdown of TNFAIP6 in GC cell repressed PTX3 expression while this effect is attenuated by PTX3 overexpression plasmid (OE-PTX3). As expected, PTX3 reversed the phenotypes observed in the TNFAIP6-suppressed GC cell. All these findings disclose that TNFAIP6 regulates GC cell invasion is partially dependent on PTX3.

### 4.5. Higher TNFAIP6 Expression Is Associated with a Poor Prognosis in Patients with GC

Finally, using The Cancer Genome Atlas (TCGA) was used to detect the prognostic value of TNFAIP6 expression in patients with GC [25]. Consistently, high TNFAIP6 expression is associated with shorter overall survival for patients with GC, as shown in Figure 6. Correlation analysis by Spearman's rank correlation coefficient show that PTX3 is positively correlated with TNFAIP6 expression in the GC. Finally, the role of TNFAIP6 on GC cells metastasis is confirmed by in vivo lung metastasis models. The mice in the sh-NC group have more and larger lung metastatic nodules, whereas fewer and smaller metastatic nodules are observed in mice injected with sh-TNFAIP6-transfected SGC7901 cells. Overall, these findings imply that knockdown of TNFAIP6 represses the metastasis of GC cells in vivo.

## 5. Conclusion

In summary, TNFAIP6 plays a critical role in cell growth, invasion, and induced EMT phenotype of GC cells. A high level of TNFAIP6 in GC tissues is related to the unfavorable prognosis of patients. TNFAIP6 overexpression increases *β*-catenin levels in nuclei and activates the Wnt/*β*-catenin signal. Mechanistic analysis revealed that TNFAIP6 increases malignancy by enhancing PTX3 expression and PTX3 has a critical role in TNFAIP6-mediated regulation of GC cell invasion and EMT.

## Figures and Tables

**Figure 1:** High expression of TNFAIP6 in GC tissues: (a) the TNFAIP6 expression levels in 31 pairs of GC tissues and the matched paracancerous tissues are measured by qRT-PCR (^*∗∗*^*P* < 0.01 compared with paracancerous), (b) the analysis of TNFAIP6 expression in paracancerous and GC tissues, (c) the patients are divided into high and low TNFAIP6 expression groups according to the scoring of immunohistochemical staining, (d) TNFAIP6 mRNA expression levels are determined using qRT-PCR in GC cells and GES-1 (^*∗∗*^*P* < 0.01 compared with GES-1).

**Figure 2:** TNFAIP6 knockdown inhibits GC cell growth and invasion: (a) the immunoblots indicate protein levels in si-TNFAIP6 transfected GC cells, (b) the Cell proliferation analysis for TNFAIP6 siRNA vs si-Con in GC cell, (c) the assays for cells transfected with si-Con or si-TNFAIP6, (d) alterations in the invasion ability of GC cell following si-Con or si-TNFAIP6 transfection. (^*∗∗*^*P* < 0.01 compared with si-Con).

**Figure 3:** TNFAIP6 overexpression enhances GC cell growth and invasion: (a) overexpression of TNFAIP6 is confirmed by immunoblotting, (b) the clone formation assay is performed using TNFAIP6 overexpressed MKN45 cells s, (c) the invasion assay on the effect of TNFAIP6 overexpression on HCT116 cell invasion (^*∗∗*^*P* < 0.01 compared with vector).

**Figure 4:** Overexpression of TNFAIP6 promotes EMT in GC cells: (a) the overexpression of TNFAIP6 decreased the E-cadherin expression and raised the N-cadherin expression, (b) the TOP/FOP luciferase activity assay on TNFAIP6 overexpression of the Wnt/*β*-catenin pathway (^*∗∗*^*P* < 0.01 compared with vector), (c) the TNFAIP6 increased the nuclear translocation of active *β*-catenin in GC cells, (d) Coexpression regulatory network obtained from the String database, (e) changes in TNFAIP6 expression on the mRNA level of PTX3 in GC cells.

**Figure 5:** PTX3 mediates the prometastatic effect of TNFAIP6 in GC (a) the SGC7901 or MGC803 cell is cotransfected with TNFAIP6 siRNA and PTX3 overexpression plasmid (OE-PTX3), (b) the clone formation assay is based on cotransfected GC cells, (c) the invasion assay based on cotransfected GC cells(^*∗∗*^*P* < 0.01 compared with vector and ^##^*P* < 0.01 compared with si-TNFAIP6).

**Figure 6:** Patients with a high TNFAIP6 expression level exhibited a poor prognosis: (a) the Kaplan–Meier survival curve of TNFAIP6 gene in GC generated from Kaplan–Meier plotter, (b) the correlation analysis for TNFAIP6 and PTX3 from TCGA database, (c) the representative images of mice intravenously injected with sh-TNFAIP6-transfected SGC7901 cells and H&E staining of the metastatic nodules in the lung, (d) the quantitative analysis of the pulmonary metastatic modules(^*∗∗*^*P* < 0.01 compared with sh-NC).

**Table 1:** The clinic pathological parameters in patients with GC.

Variables	Cases (*n*)
Age (years)	
≤50	9
>50	25
Gender	
Female	11
Male	23
Tumor stage	
I-II	30
III	4
Metastasis	
Negative	24
Positive	10

## Data Availability

The simulation experiment data used to support the findings of this study are available from the corresponding author upon request.
